The article "Deep-Learning-Based Cancer Profiles Classification Using Gene Expression Data Profile" was published in 2022. Journal: J Healthc Eng.

# Deep-Learning-Based Cancer Profiles Classification Using Gene Expression Data Profile

**DOI:** 10.1155/2022/4715998

**Published:** 2022-01-07

**Authors:** Hatim Z Almarzouki

**Affiliations:** Department of Radiology, Faculty of Medicine, King Abdulaziz University Hospital, Jeddah, 21589, Saudi Arabia

## Abstract

The quantity of data required to give a valid analysis grows exponentially as machine learning dimensionality increases. In a single experiment, microarrays or gene expression profiling assesses and determines gene expression levels and patterns in various cell types or tissues. The advent of DNA microarray technology has enabled simultaneous intensive care of hundreds of gene expressions on a single chip, advancing cancer categorization. The most challenging aspect of categorization is working out many information points from many sources. The proposed approach uses microarray data to train deep learning algorithms on extracted features and then uses the Latent Feature Selection Technique to reduce classification time and increase accuracy. The feature-selection-based techniques will pick the important genes before classifying microarray data for cancer prediction and diagnosis. These methods improve classification accuracy by removing duplicate and superfluous information. The Artificial Bee Colony (ABC) technique of feature selection was proposed in this research using bone marrow PC gene expression data. The ABC algorithm, based on swarm intelligence, has been proposed for gene identification. The ABC has been used here for feature selection that generates a subset of features and every feature produced by the spectators, making this a wrapper-based feature selection system. This method's main goal is to choose the fewest genes that are critical to PC performance while also increasing prediction accuracy. Convolutional Neural Networks were used to classify tumors without labelling them. Lung, kidney, and brain cancer datasets were used in the procedure's training and testing stages. Using the cross-validation technique of k-fold methodology, the Convolutional Neural Network has an accuracy rate of 96.43%. The suggested research includes techniques for preprocessing and modifying gene expression data to enhance future cancer detection accuracy.

## 1. Introduction

With increasing data dimensionality in machine learning, the quantity of data required for analysis grows exponentially.

Bellman alluded to the “curse of dimensionality” while acknowledging the challenges of dynamic optimization. The issue is solved by projecting a high-dimensional dataset onto a smaller variable number (or feature) that preserves the information. Microarray data usually pertain to a small sample issue. Each data point (or sample) may include up to 450,000 variables (gene probes), resulting in a significant computational cost. Due to the sparsity of such relevant data for every dataset, it is very difficult to show that this finding is statistically significant. Large datasets with a “large *p*, small n” issue (where *p* is the number of features and *n* is the number of samples) may lead to overfitting. The difficulty may arise due to loud characteristics.

The article "Deep-Learning-Based Cancer Profiles Classification Using Gene Expression Data Profile" was published in 2022. Journal: J Healthc Eng.

Gene expression data have been found to be both data-rich and data-poor in terms of information, and the public databases of the microarray are the National Center for Biotechnology Information, GenBank, the Array Express, the Gene Expression Omnibus, and the Stanford Microarray (NCBI, GenBank, Array Express, Gene Expression Omnibus, and Stanford Microarray).

Microarrays provide genome-wide patterns in gene expression, increasing the clinical uses of this technology for illness diagnosis, therapy, and prognosis.

WPact features [1]. On the basis of several molecular or genetic investigations, it is possible to enhance the survival rate of cancer patients following a cancer diagnosis by using a wide range of medications. According to the findings of the study, early identification and therapy may be enhanced by minimizing the adverse effects associated with the treatment. The study of impaired gene expression in cells is used to determine the characteristics of carcinogens. The gene expression data from tumor cells are collected using a microarray, which provides a significant amount of information for the research process and may be utilized to guide future studies. The dataset contains hundreds of distinct gene expression profiles, each of which has precise feature values and may effectively analyze mechanisms [2]. This dataset also includes the gene expression recommendations, which can be accessed here. Several previous researches used deep learning and machine learning to detect cancer types using microarray gene expression and a normal subset of genes. The impending work comprises a preprocessing stage, which is a normalizing phase that helps to reduce training time. Feature selection methods are important in gene expression data analysis for cancer classification [3] because they assist in reducing data dimensionality. The reduced dimension may affect the biomarker method. The feature selection technique may be used to eliminate noisy features early on [4]. It is feasible to describe biological features while reducing model complexity by reducing feature complexity during feature selection. Unsupervised learning may assist to improve tumor profiles by enhancing certain gene features during segmentation.

The article "Deep-Learning-Based Cancer Profiles Classification Using Gene Expression Data Profile" was published in 2022. Journal: J Healthc Eng.

Latent [5] characteristics are selected from the auto-encoder procedure. Among the characteristics retrieved during feature extraction is the training procedure's separation of tumor kinds and subtypes. This study's unsupervised method is the most important since it can pick genetic factors without the use of tumor markers; derived from clinical data combined with high-dimensional gene expression data from lung, kidney, and brain tumors, the proposed unsupervised feature selection method is used to pick features [6]. Microarray technology is currently considered to be a critical tool for scientists who want to monitor the expression of genes in a living organism. Microarray technique uses a glass plate on which DNA molecules are fixed in an ordered way. As illustrated in Figure 1, characteristics are linked to each gene in the dataset.

There may be hundreds of these places on the microarray, each containing about a million copies of the undistinguishable DNA molecules linked with the gene. In the location, any gene will identify genomic DNA, or a short oligonucleotide strand modified to match any gene as DNA. Microarrays have been used for the appearance of the gene in various ways and continued in a particular condition (state A) for a comparable collection of genes from reference cells (state B). Figure 1 depicts the overall picture of these first movements. To differentiate between the two transcriptions, RNA from cells is first extracted, and then reverse transcriptase is used to turn it into cDNA.

Allow cDNA from state A cells to be examined with one red dye and cDNA from state B cells to be analyzed with a green dye. They will hybridize to the exact locations on a glass slide that has a similar arrangement of the same kind if they are marked differently. When cDNA is attached to a spot, the actual quantity of cDNA is proportional to the original number of RNA molecules and the number of molecules of the gene present in the samples.

These areas in a hybridized microarray will be stimulated using a laser and scanning at their proper wavelengths for detecting the red and green dyes, respectively, after completing the processes.

The quantity of fluorescence produced upon excitation will be proportional to the amount of nucleic acid that has been bound. As a result, if a cDNA with condition *X* in a specific gene is in profusion from condition Y, the spot will be reflected as red in the cDNA. Otherwise, the color will be green. If the gene has been expressed in a similar manner, the spot may be yellow, and if the gene has not been expressed, the area may be completely black. Consequently, for each place on the microarray belonging to a gene, there will be an associated value of fluorescence, which will be displayed as the gene's expression level in the picture of the array.

The article "Deep-Learning-Based Cancer Profiles Classification Using Gene Expression Data Profile" was published in 2022. Journal: J Healthc Eng.

Using the principles of nucleic acid hybridization and pairing, the Microarray technology has been developed to identify seven such complementary sequences in compound combinations. Single-stranded labelled “probes” of all of the recognized sequences have been developed to detect the presence of unknown samples and their compliments on the microarray. The early techniques of macroscopic hybridization are employed as flexible and porous filters to provide a solid support for halting the detection probes, which are used as solid supports for stopping the probes. This starting use of solid supports such as glass and the decrease of all of the immobilized nucleic acid characteristics that were apparent as soon as the first microarrays appeared were all significant developments.

The “probe” refers to the immobilized strand in the nucleic acid, and the “target” refers to a complimentary phase component that is used in conjunction with the “probe.” For the most part, the probes on the microarrays were of three kinds. The first was cDNA, the second was resynthesized oligonucleotides, and the third was in situ synthesized oligonucleotides (also known as in situ synthesized oligonucleotides). The novelty and the major contribution of the proposed work in the identification of informative genes are accomplished by statistical metrics or optimization strategies. The marker genes utilized in this study were selected using a two-step procedure. The initial stage involves retrieving feature subsets from the database. The first phase involves analyzing the original microarray data with statistical measurements, and the second step involves analyzing the original microarray data with statistical measures. Look for the optimum feature subsets that will enhance the classification performance. Heuristic optimization is used to improve performance. Heuristic optimization is used to improve performance. The organization's fundamental goal is to The purpose of the study is to find the marker genes that increase categorization accuracy. The goal of the study was to find the marker genes that increase categorization accuracy.

The following is the structure of the paper.  Section 2 contains examples of related work, while Section 3 contains information on materials and techniques.  Section 4 of the planned task is an investigation.  Section 5 contains the findings and conclusions of the planned research project. Section 6 of the planned work covers the completion of the work.

## 2. Background Analysis

There are several surveys relevant to the planned work that is being conducted by different research organizations. As a result of the feature selection method, Ang et al. [7] found the dimensionality of gene expression data may be according to the American Cancer Society; the subtypes of colorectal cancer have been characterized by their latest molecular classifications in terms of global gene expression.

The article "Deep-Learning-Based Cancer Profiles Classification Using Gene Expression Data Profile" was published in 2022. Journal: J Healthc Eng.

According to the American Cancer Society, the subtypes of colorectal cancer have been characterized by their latest molecular classifications in terms of global gene expression. Summary: They are displaying opposition to therapy, in addition to other signs of opposition. In order to avoid an erroneous assessment of the situation, several categories have been examined, and a decision has been reached. Erroneous assessment of the situation Several categories have been examined, and a decision has been reached by Calon et al. (2015) [8] found that it is via the genes represented through the chromosomes; It is stromal cells, not epithelial tumour cells, that can predict the future. It is the stromal cells, not the epithelial tumor cells [9], which can predict the future. There has been a relapse of the illness across all classifications. Linked with bioinformatics and immunological responses to chemical analyses in the pharmaceutical industry, identifying stromal markers has been shown via functional investigations that Cancer-Associated Fibroblasts (CAFs) are responsible for increasing the frequency of cells that start this tumor. This frequency may be raised significantly by altering the environment. The signaling of the Growth Factor beta (TGF-beta). Gene software that has been developed using TGF-beta-induced stromal cell proliferation in tumors is associated with a poor prognosis. CRC subtypes are linked with each other. It has been shown that the usage of TGF-beta signaling inhibitors, which block the production of TGF-beta, may prevent illness. This medication prevents cancer cells from communicating with one another and with the surrounding environment. Tumor organoids and xenografts generated from human tumors may be used to detect [10] cancer patients.

A promising and novel method for identifying cancer and metastasis has been developed. The most recent advances in construction and architecture have given opportunities for metastasis. In addition, dynamic bimolecular settings for different cancers are being investigated. Types: as a result, we may assume that the connections between gene expressions are significant. By studying different types of cancer, we may have a better understanding of how cancer develops early on in bimolecular networks that have been linked to both normal and pathological processes. Cancerous states are a kind of cancer. This theory has been tested by Ling et al. (2014), and they investigated if there is a relationship between the mRNA terminologies of three different genes.

The article "Deep-Learning-Based Cancer Profiles Classification Using Gene Expression Data Profile" was published in 2022. Journal: J Healthc Eng.

When the cancer-related genes PIK3C3, PIM3, and PTEN were randomly selected, “The cancer had advanced,” and these coefficients have been put through their paces in the field of cancer research. Diagnosis: during the course of the illness, the following observations were made: it was discovered that there were robust correlations (0.68 r 1.0) between the variables: PIM3 and PIK3C3 in breast cancer; PIM3 and PTEN in breast, renal, and ovarian cancer; and malignancies of the liver and thyroid, and cancers of the breast and ovary involving PIK3C3 and PTEN cancers. This ascribes that the connections for early cancer diagnosis are important for the gene expression profiles of cancer networks and may be added to the current clinical data. Biomarkers such as cancer antigens are examples of biomarkers. Cancer is responsible for about ten to fifteen percent of all human deaths. Viruses: to discover novel viruses and the relationships that exist between them, massive parallel sequencing has shown to be effective in both malignant and normal tissues.

In certain patient populations, this approach has not yet been implemented. An example from Tang et al. (2013) [11] has utilized additional data from The Cancer Genome Atlas Research Network. More than 700 billion transcriptome sequencing reads were generated, and various kinds were tested. Human malignancies comprise 44 tumors and nineteen cancer types for those acquainted with them and new viruses. The present state of knowledge has been verified and improved by the map created due to fusion events with the human papillomavirus (HPV) occurring regularly. Insertions were found in the RAD51 B and ERBB2 genes. The allusions to the patterns of co-adaptation between the papillomavirus oncogene and the host are responsible for the virus's function. Gene expression in both the host and the virus genome to construct the framework of a point of reference for future research on tumor-associated viruses and a virus-tumor association with the use of transcriptome sequencing was proposed to create a map on an unexpected scale. Data: Song and colleagues (2012) [7] carried out population-based training in LINQ, China, to determine the effectiveness of serum miRNAs as biomarkers for early detection of cancer; gastric Cancer may be detected early (GC). Subjects were selected from two major training groups. Differential miRNAs were selected and analyzed using the TaqMan low-density array; they were detected in serum pools from both GC and control subjects. These were proven in a study—they were individually selected from eighty-two pairs of GC and control subjects and forty-six pairs of dysplasia participants.

The article "Deep-Learning-Based Cancer Profiles Classification Using Gene Expression Data Profile" was published in 2022. Journal: J Healthc Eng.

The real-time quantitative reverse transcription-polymerase chain reaction was used to monitor and regulate the process. Furthermore, in previous research, 58 GC patients were included. Prior to the GC diagnosis, at least one blood sample must be collected, as a progressive, to believe in a brighter future. The discovery of new advancements in known serum miRNA expression has continued. Based on the results of a long-term follow-up with a group of individuals, the serum samples that were obtained were collected over a period of five years before the clinical diagnosis of GC was determined. According to the panel, the total accuracy rate was 79.3 percent. As a result, it was shown that these three serums showed their promise as novel diagnostic tools for the early identification of GC noninvasive biomarkers.

Allory et al. [12] found that stimulating the expression of the genes was effective (2014); the promoter of gene coding has documented and suggested hotspot modifications for the transcription of a gene sequence. Telomerase reverse transcriptase is an enzyme that helps to lengthen the lifespan of cells (TERT).

The following may be investigated further:

Aspects of Urothelial Bladder Cancer's (UBC) spectrum, its relationship to expression and clinical prognosis, and the prevalence of TERT mutations to assess the TERT To study promoter alterations, a cohort of 111 UBCs at various phases of development was used. Sequencing using the Sanger method and messenger RNA (mRNA) communication via TERT, the reverse transcription-quantitative polymerase chain reaction was used to accomplish this Using the Snapshot test, the two most frequently occurring mutations have been identified. UBC researchers examined a separate group of 184 non–muscle-invasive and 173 muscle-invasive UBC patients. Bennet et al. (2014) [13] propose a hybrid approach for evaluating and classifying microarray data, and it was based on SVM, Nave Bayes, and other techniques. It was used to classify microarray data, and it was based on SVM, Nave Bayes, and other techniques. KNN: before any other consideration, feature selection is a very essential classification. The method of feature selection links Discrete Wavelet with a particular characteristic. The double-wave transform (DWT) and the moving window technique (MWT): the proposal is as follows: the presentation of the method has been evaluated against conventional classifiers like Support Vector Machine, Naive Bayes, and KNN, which are all examples of machine learning algorithms. The experiments' results have shown that the ensemble method is more effective in getting results. When compared to traditional methods, classification accuracy [14] is much higher. This study, which serves as an automated method for cancer categorization, is noteworthy. Doctors have a sense of security. It also has the additional benefit of lowering the likelihood of making a mistake. Cancers are classified according to their location. A single or a combination of gene expression changes has been authenticated. A “gene expression signature” is a term used to describe the specificity of a gene expression profile [15]. This has been verified. Using prognosis, diagnosis, or the prediction of treatment response as a starting point, however, because of the case's appeal, the rules of evidence must not be disregarded. This molecular method, as well as discovery-based research, has the potential to lead to erroneous assertions. The following authors have addressed these fundamental issues: Chabon (Japanese for “chicken”) is a kind of pigeon that is native to Japan (2013) [16]. He has also provided proof of the effects on both a biological and a psychological level. Clinical levels are referred to as several studies that have shown that this gene expression profile is accurate.

The article "Deep-Learning-Based Cancer Profiles Classification Using Gene Expression Data Profile" was published in 2022. Journal: J Healthc Eng.

It is more successful in improving our knowledge of cancer biology. It can predict the development and reaction of the disease and the capacity to monitor the cure of cancer. The probability of finding a shared diagnostic biomarker for two diseases Cancer of Unknown Primary (CUP) was investigated using a microarray gene expression analysis in the Kobayashi et al. (2013) [17] research work, and they have proposed an exemplary method of analysis. The Affymetrix is a statistical method. For the analysis of tumor mRNA samples, the U133 A plus 2.0 Gene Chip was used. From a group of about sixty individuals with CUP, Asin (hyperbolic arcsine) to formulate a mean, the transformation was performed to normalize the data. A gene-expression profile exclusive to CUP Microarray datasets in their raw form was made accessible to the public to construct a gene expression profile which is also true, especially for the non-CUP group. This is especially true for the non-CUP group. The CUP and the non-CUP parties have negotiated a settlement. The *t*-tests have been used to compare two groups of data. The CUP genes in the top fifty-nine positions have the. It was decided to choose the maximum fold with a probability of less than 0.001. Six points out of ten in the set of the forty-four genes that were found to be upregulated in the CUP set were classified, and ribosomal proteins [18] are proteins found in ribosomes. RPS7 and RPL11 are two genes that are members of the RPS7 gene family. The Mdm2–p53 pathway is involved. By suggesting that the CUP has a biological characteristic, many genes have been identified as being related to metastasis and apoptosis.

The article "Deep-Learning-Based Cancer Profiles Classification Using Gene Expression Data Profile" was published in 2022. Journal: J Healthc Eng.

Following the feature selection of molecular data, the suggested method has been related to the triple-negative breast cancer subtype. However, this method is not accurate because of the unsupervised job given to the trainees throughout the training phase. During the feature selection process, the proposed study explains how to overcome the limitations of unsupervised learning. The method of extracting multi-selection features from microarray data is characterized as an unsupervised training procedure based on the data. This method is used based on the weights assigned to each component acquired during the data partitioning process and the subset of features generated. However, one of the disadvantages is that weight loss occurs throughout the L1 normalization process. This paper proposes classification methods based on unsupervised learning and feature selection strategies based on the normalization of gene expression for use during classification [19]. The input dimension may be decreased using the Latent feature extraction method, which is used in conjunction with the selection of gene expression characteristics using the latent representation technique.

## 3. Proposed Methodology

The proposed work consists of two main stages, namely, training and testing stages. During the training stage of gene expression data, feature selection is carried out to categorize the input gene expression dataset.

Machine learning methods provide a solution to the issue of having a large number of datasets to work with. The data may be split into two categories: the training dataset and the validation dataset, respectively. This data collection is used to calibrate the parameters of certain models that have been developed using it. The training dataset is used to evaluate the effectiveness of the learned features. The Kaggle gene expression dataset is used to collect data and it is an open dataset that is available for the researchers to access freely and identify the cancer using machine learning algorithm.

This paper [20] suggests that one of the unsupervised learning techniques, known as the Latin structure method produced from autoencoders, should be referred to as a reference in the future. It must go through three stages to complete the planned task: feature selection, training, and testing. Based on the latent space, target kernel matrix ring samples are generated.

The article "Deep-Learning-Based Cancer Profiles Classification Using Gene Expression Data Profile" was published in 2022. Journal: J Healthc Eng.

Figure 2 represents the flowchart of the proposed work. The characteristics that have been chosen go through their categorization procedure to categorize the different kinds of cancer. It is common practice to utilize microarray categorization to distinguish between genes for the purpose of identifying different tissue types, which is particularly helpful in the diagnosis of cancer. The introduction of machine learning methods has aided in the systematic exploration of DNA microarray gene expression data, allowing for higher throughput research than was previously possible using histology techniques. Microarray data with high dimensionality generated from limited sample numbers, on the other hand, is a significant problem that must be addressed [21]. In most cases, just a few hundred tissue samples are needed to generate tens of thousands of gene expression profiles. The use of feature selection techniques to deal with high dimensionality has become the standard to overcome this problem.

The feature selection method identifies the suitable features. It discards the inappropriate elements, resulting in a reduction in the input dimensionality and an improvement in the classification performance of the classifier. Furthermore, many studies have shown that most genes discovered via DNA microarray study are insignificant for making an accurate difference between different classes of the issue. To avoid being plagued by the curse of dimensionality, feature selection is an essential component of DNA microarray research. The second important rationale for reducing dimensionality is that it will aid scientists in discovering the underlying mechanism that links gene expression to disease progression.

In data mining, feature selection is used in a number of different fields such as classification, association rules, clustering, and regression. Feature selection algorithms developed using a variety of evaluation concepts may be divided into three categories: filter algorithms, wrapper algorithms, and hybrid models. Without taking into account any mining method, the filter model is based primarily on generic characteristics of the data analyzed, and feature subsets are chosen without taking into account any mining process. Searching for more suitable features for mining algorithms is more time-consuming than searching for features that are better suited for other algorithms. The hybrid model makes use of the advantages of both models by using both of their changed assessment criteria at different search stages, thus maximizing their combined benefits. To divide each point, machine learning algorithms choose the most relevant characteristics to the situation at hand; ideally, one should never pick unnecessary or redundant traits. It is widely accepted that the addition of irrelevant characteristics to a dataset “confuses” the machine learning system in situations when there is overfitting and makes the system less understandable [22].

The article "Deep-Learning-Based Cancer Profiles Classification Using Gene Expression Data Profile" was published in 2022. Journal: J Healthc Eng.

In a document, information gain (IG) is defined as the quantity of information gained for the purpose of making a group prediction. The existence vs lack of a feature is used to evaluate the reduction in entropy in a system. This application may be thought of as a generic method that assesses informational entropy to determine a specific characteristic's significance. When combined with Shannon entropy, informational entropy may be used to calculate the amount of data needed to encode a particular piece of information. The entropy of a system is directly proportional to the amount of space taken up by the information it is trying to encode.

When it comes to categorization, the information at stake is the distribution of instances inside different classes of objects. If the instances are allocated haphazardly among classes, the number of bits required to encode this class distribution is large since each individual example must be calculated. When all of the instances are members of a single class, the entropy is reduced. Consequently, when the class distribution is spread in a large number of subgroups, the entropy of subsets of the data should rise, according to the entropy-measurement function.

The murmur is a feature selection technique in which features are chosen based on their high correlation with the class (output) and their low correlation with one another (internal correlation). In the case of continuous features, the F-statistic is used in the calculation of the correlation between features (relevance) and the computation of the correlation between features and other variables (redundancy). It is necessary to apply the Pearson correlation coefficient. The features are selected one by one using a greedy search to maximize the objective function, which may be thought of as a function of relevance and redundancy. The selection of features is made in this manner: one feature is selected after another.

In this study, the objective functions that were utilized were the Mutual Information Difference (MID) criteria and the Mutual Information Quotient (MIQ).

As represented in Figure 3, the preprocessing stages consist of histogram values, mean, and standard deviation calculation, which would eliminate the noisy data in the input dataset. When using the feature selection method, certain preprocessing procedures are needed since the approach flattens temporal data into a single matrix, which results in a loss of information among the temporal data.

The article "Deep-Learning-Based Cancer Profiles Classification Using Gene Expression Data Profile" was published in 2022. Journal: J Healthc Eng.

When the relief algorithm assigns relevance weights to each characteristic, it takes advantage of instance-based learning to do so. Weights are allocated to each feature among the many class values. A final subset of characteristics is produced by ranking the features according to their weight and selecting the higher weight features than the user requested. Threshold: in this approach, training data examples are selected at random from a pool of instances. Upon sampling a feature, the closest feature of the same and opposite class is identified for that feature. The weight of an attribute is updated depending on how its values are differentiated from those of the sample features and those of its closest hit and miss neighbors, respectively. The importance of a feature increases if it differentiates between characteristics from distinct classes while maintaining a consistent value for features from the same class.

According to the importance of the feature relief algorithm to the classification job, an algorithm is given to each feature relief feature. Initially, all weights are given a value of zero, and then 50 iterative updates are carried out. During this procedure, two groups of instances are selected: those with the closest characteristics that belong to the same class, and those with a distinct set of features that belong to a separate class. Relief-F is used to deal with multi-class issues since it expands Relief's capabilities to allow for dealing with incomplete and noisy information.

Relief-D is a deterministic version of the algorithm that uses all occurrences and the near-miss and near-hit of each feature. This results in the equivalent running relief being available for an indefinite period of time after that.

The disadvantage of univariate filters, such as IG, is that they do not account for correlations between features, which may be reduced by multivariate filters, such as Correlation-based Feature Selection, which is described below (CFS). The value of a subset is determined via the use of CFS of attributes, which considers the individual predictive power of each feature and the degree of redundancy among the characteristics. It is possible to estimate the correlation between subsets of features and class and the correlation between features themselves using the correlation estimate. When there is a connection between features and classes, the significance of a set of features increases and declines as the intercorrelation between features and classes increases [19]. CFS aids in the determination of the optimal feature subset and is often used in conjunction with other search methods such as forward selection, bi-directional search, backward elimination, best-first search, and genetic search to get the best results.

The article "Deep-Learning-Based Cancer Profiles Classification Using Gene Expression Data Profile" was published in 2022. Journal: J Healthc Eng.

### 3.1. Dataset

Each patient's data point was collected via the use of microarrays, and this dataset is a collection of those data points. The data collection includes high-dimensional gene expression information obtained from a range of tumor profiles, and the information is organized into categories. Cancers such as lung cancer, kidney cancer, and brain cancer are among those that may be discovered. To get information about cancer genome quotes, you must first visit the global cancer genome quotation site. 840 and 345 cancer samples from the squamous cell subtype and adenocarcinoma subtype, respectively, are mixed up with cells from the adenocarcinoma subtype in the lung cancer dataset [23]. With 145 and 439 samples, respectively, in each category, the brain cancer dataset may be split into two types: benign and malignant forms of brain cancer. The papillary renal cancer dataset has 320 tumor samples, whereas the clear cell renal cancer dataset contains 260 tumor samples. The datasets are split into two groups. The number of cancer samples is given by *n*, and the number of protein-coding genes in each dataset is given by dm. The data matrix of each dataset is denoted by the notation Un, dm (uniform data matrix). P must be less than dm to choose a subgroup; *p* denotes the gene normalization process.

Table 1 summarizes the dataset collected from different databases, including patient recordings. The sample dataset includes both normal and infected patient samples.

### 3.2. Preparation of Dataset

For the experimental methods, it is possible to split the data into two groups. The first group contains the feature X1; the second group has the sir classes X2. The matrix value is structured as main underclass nx1, where x represents the number of samples and n indicates the number of genetic factors in each class in the feature matrix of the feature. The data collection, which contains a variety of samples, is split into two parts: training data and authentication data. The training samples consist of 139 models, whereas the authentication samples consist of 36 models each. The training dataset is used to perform the first calibration, which is done using a deep learning algorithm with the training dataset. The hyper parameter was applied to the validation set and is used to determine the correctness of the algorithms in question. The correctness of each procedure is determined by adjusting the hyper parameter using the fold cross-validation method to prevent overfitting the values [24, 25]. The datasets utilized in the future study have a greater dimensionality than the original datasets. The direct application of a dataset may impact the accuracy and outcomes based on dependability and consistency. The normalizing method is included in the preprocessing step to address this issue. During model training, normalization may aid in the reduction of noise and the improvement of imperfect relevant features. To decrease the size of the feature components from 12633 to 133, the PCA method is utilized to perform normalization.

The article "Deep-Learning-Based Cancer Profiles Classification Using Gene Expression Data Profile" was published in 2022. Journal: J Healthc Eng.

### 3.3. Initial Stages of Processing

#### 3.3.1. Data Analysis: Preprocessing

The read count value of gene expression is included inside the dataset. The range of gene expression fluctuates and is less than one in size. This means that the logarithmic equations must be used to perform the transformation:

(1) $$\begin{array}{c} x=\;\log_{2}\left(y+1\right). \end{array}$$

If the values are less than one, (1) will decrease the grading appearance based on the standards that are less than one to zero, thus reducing the scaling expression. With the normalization technique, it is possible to remove 1000 genetic expression [26] levels that were found because of noise added gene values. The variable *x* represents the gene characteristics acquired from the microarray dataset in calculation 1, which signifies the gene characteristics received from the microarray dataset. With the usage of filtering techniques, the threshold value will be the same as 1.19 in the gene expression throughout the whole sample when the filtering methods are used. Depending on the threshold setting, the accuracy and consistency of classification are both compromised. Because the lower threshold value preserved a greater number of genes, the value of a specific biomarker will not be reduced. It is possible to convert normalized values into gene expression levels by using input genitival microarray representation, as the third phase begins with the transformation that was used to estimate the performance of the intended job. This is the beginning point for the fourth step. Asymmetrical transformations are applied to the data, which are determined by the properties of the individual datasets. When it comes to passing the suggested job, the Latent Feature Assortment Technique is employed, and the feature assortment procedure is essential for accomplishing the given task (LFST).

When using the recommended feature selection approach, the latent feature selection methodology is used to pick the most relevant features. It is composed of *m* growth examples with the typical d1 gene appearance topographies in the matrix range of Amd1 and the latent feature selection method, which are used in conjunction with the d1 gene appearance features. In the case of regularized topographies with a lower range, the form of *p* is represented in the case of d1, while the form of *p* is represented in the case of d2. Initially, the trained feature is produced via the use of an autoencoder model in combination with the PCA feature extraction technique. This trained feature is then used as the starting point for the feature selection procedure. It is necessary to train the Convolutional Neural Network on the features retrieved via PCA before using it to perform the feature selection process on the features. When the latent space is stated in the form of the *z* dimension, the latent space meets the criteria ld. A Latent space with a Gaussian kernel was used to project the Amd1 data in order to get the final outcome in this case. In the Gaussian kernel emulator, the Gaussian kernel is represented by the symbol KZ and utilized as a target kernel. A kernel for each feature is created by constructing Amd1, the matrix holding the D1 set of features. This results in the creation of a kernel for each feature in D1. Finally, the most recent model is used to reduce the subset of *p* centers that are alternately designated and merged to create K with an upsurge in the arrangement of the kernels in the matrix, with an increase in the arrangement of the kernels in the matrix.

The article "Deep-Learning-Based Cancer Profiles Classification Using Gene Expression Data Profile" was published in 2022. Journal: J Healthc Eng.

Figure 4 depicts a diagrammatic representation of the planned technique. Using this technique, a sparse key is produced, in which the existence of nonzero standards of the course indicate the presence of unique importance at the consequence. Using an unmanaged method, the features are selected in a way that is very well matched with the representation produced by the auto encoder. To describe this method, we have coined the name, “Latent feature selection technique” (LFST).

#### 3.3.2. Stage 2: Selecting the Best Feature from the Input Dataset

The Latent Feature Selection Method consists of an optimization procedure that inputs the normalized score features collected and utilizes them to choose the most suitable components. The feature selection process is organized using an unsupervised approach, and the best features are selected using the procedure results. It is necessary to utilize an m-dimensional interplanetary purpose value that is symmetrical and semi-positive to meet the criterion.

(2) $$\begin{array}{c} k\left(x_{i},x_{j}\right)=\phi \left(x_{i}\right),\phi {\left(x_{j}\right)}_{H}. \end{array}$$

Here, apply the Hilbert space transform, where the purpose signifies the dimensionality of the high-dimensional information and H is the Hilbert interplanetary convert coefficient shown in equation (2). The Hilbert interplanetary transform is defined as the head of the matrix dimension of the function H operations in a couple of single vector values in Hilbert space multiplied by the number of operations in the Hilbert space transform. The Hilbert space transformation is another name for this transformation. The labelled samples may be represented visually in equation (3) by the number of labels:

(3) $$\begin{array}{c} \phi :X\mapsto \phi \left(X\right)\in ℋ. \end{array}$$

It is represented by (3) and defined as *X*_i_, the kernel matrix obtained, which may be regarded as information for the training phase.

(4) $$\begin{array}{c} k\left(x_{i},x_{j}\left\{\left(x_{1},y_{1}\right),\left(x_{2},y_{2}\right),\ldots ,\left(x_{n},y_{n}\right)\right\}\right)=\phi \left(x_{i}\right),\phi {\left(x_{j}\right)}_{H}, \end{array}$$

where *n* is the number of characteristics that were present in the genetic factor sample collection; the kernel may be constructed using a function derived from the core matrix, which produces the desired output.

(5) $$\begin{array}{c} \text{Amdl}=\phi \left(x_{i}\right),\phi \left(x_{j}\right)=k\left(x_{i},x_{j}\right). \end{array}$$

Equation (6) provides the matrix form of the characteristics that have gathered the information. When the output is expressed in binary form, the samples are different and comparable.

(6) $$\begin{array}{c} k\left(x_{i},x_{j}\right)=\exp\left(-\gamma x_{i}-x_{j}^{2}\right). \end{array}$$

Various kernels are available. K1 and K2 both have different numbers of samples, as well as different arrangements of the board. The sample set has a variety of topographies that may be used for preparation, and it is composed of three regulated input appearances. Equation (7) signifies the two tested dataset ethics with regulated structures as represented by the two sampled dataset values. It is possible to compare two kernels with sample set *M* by using the alignment method.

(7) $$\begin{array}{c} A\left(K_{1},K_{2}\right)=\frac{K_{1},K_{2F}}{\sqrt{K_{1},K_{1F}K_{2},K_{2F}}}. \end{array}$$

Element selection is made out using equation (8) to separate the characteristics that can be utilized in the keeping fit and challenging phases of classifiers [20] to evaluate the different classes from those that cannot.

(8) $$\begin{array}{c} K_{\mu }\left(x,x^{\prime }\right)=\sum_{i=1}^{n}\mu_{i}K_{i}\left(x,x^{\prime }\right),\mu_{i}\geq 0. \end{array}$$

The article "Deep-Learning-Based Cancer Profiles Classification Using Gene Expression Data Profile" was published in 2022. Journal: J Healthc Eng.

## 4. Training and Testing Results

It is necessary to incorporate the Convolution Neural Network Classifier in both the training and testing stages of the process since it is based on a deep learning method. For the prediction of specific cancer types, it has been proposed that a CNN model be used. Each CNN model is intended to perform this function in order to create gene expression, data models. Class predictions are produced based on the qualities that have been selected or arranged and have been given as input. It is necessary to employ a one-layer Convolutional matrix with restricted samples for the development of the CNN architecture. The number of parameters used in the network determines how many samples are utilized. The CNN model is built on a one-dimensional kernel with two input vectors as its foundation. Reference [25].

Figure 5 depicts the CNN model's planned architecture, as shown in the diagram. A significant difference exists between the proposed CNN classical and the commonly used CNN prototypical, which is based on the period sequence prediction, which reflects the distance of the scope of the core in the proposed CNN model. In this case, the global features relate to the initial kernel size and the Convolutional value. The suggested architecture has the potential to capture certain characteristics of gene expression. This is accomplished via the use of a cascaded connection between the activation function and the maximum pooling technique. The Convolutional module comprises a SoftMax layer that can forecast the different kinds of cancer.  Table 2 shows the input parameters of the proposed work.

The Kera's visualization package [27] was used to create the visual representation of the CNN model. More precision is achieved by using gradient classes to account for minor variations in the gene expression levels.  Figure 6 provides the training and testing epoch rate within the classifier.

The gene has a copy number of 2.6 and is classified as a cancer gene. The epoch and batch size are set at 60 and 128, respectively. Initially, all CNN models were trained on the different tumor samples that were available. Figure 5 represents the training and testing dataset of the proposed work. In this study, the over-fitting and the loss function [28] are used to assess the training process. The model incurs certain losses, which are shown in Table 3.

In Table 3, the training and testing epoch networks are used in the proposed work. The training and testing phase of a neural network requires twofold cross-validations, which may be performed three times. Classification accuracy may improve or decrease by 0.3 percent for 93.3, 93.8, and 97.1.

Figure 7 represents the model accuracy of the proposed work. The proposed accuracy is calculated from the training as well as testing phases.

One of the main flaws of microarray technology is the production of noise. Some advanced noise reduction and data normalization approaches may be investigated in addition to the suggested feature selection methods. Differentially expressed genes (DEGs) may be investigated. Statistical methods like fold-change, *t*-test, and ANOVA are often employed to identify DEGs. The use of heuristics to solve the DEG issue is possible. It is planned to include more meta-heuristic methods and improve the computational complexity. These natural optimization methods may be used with classifiers to improve classification accuracy [14].

The article "Deep-Learning-Based Cancer Profiles Classification Using Gene Expression Data Profile" was published in 2022. Journal: J Healthc Eng.

Table 4 represents the performance metrics obtained from the experimental analysis [29] of the existing algorithm.  Table 5 represents the performance metrics from the proposed work.

Figure 8 represents the performance metrics of the proposed methodology with the prediction rate. The prediction rate is analyzed from the true positive and true negative values from the training and testing data.

## 5. Conclusion

The subject features and superfluous features are suggested to be reduced from a large dimensional feature of gene expression [29] data using a feature selection method known as latent feature selection, which is also known as the latent feature selection technique. The experimental findings provide the optimum feature selection method output for achieving accurate classification based on the chosen features derived from experimental data. The categorization feature has an accuracy rating of 93.43 percent, with the smallest amount of loss possible. Cancer may be readily identified and diagnosed if it is discovered and diagnosed at an early stage. The discovery of specific medicines for early diagnosis treatment is made more accessible as a result of this. The evaluation of genetic and metabolic characteristics of different datasets will be included in future studies.

## Figures and Tables

**Figure 1:** Interconnect Information of genes in the dataset.

**Figure 2:** Flow chart of the proposed work.

**Figure 3:** Preprocessing stages of gene expression.

**Figure 4:** The suggested method's pipeline is shown in this diagram after the raw data have been processed.

**Figure 5:** Input classifier model architecture.

**Figure 6:** Training and testing graph.

**Figure 7:** Proposed architecture lost and accuracy.

**Figure 8:** Performance metrics of the proposed work.

**Table 1:** Input Datatypes of the proposed work.

Type	Subtype	Patient samples
Renal input data	Papillary	320
	Clear tumor	260
Brain dataset	Benign	145
	Malignant	439
Lung dataset	Squamous cell	840
	Adenocarcinoma	345

**Table 2:** Proposed classifier input parameters.

Input parameters allocated	Proposed classifier best
	Value analysis
Train size = 9000	Train size = 9000
Test size = 1000	Test size = 1000
nummular = 1	nummular = 0
dropout = False	dropout = False
train_valid_split = 0.5	train_valid_split = 0.5
channels = 4	channels = 32
patience = 10	patience = 10
Weight decay = 0.00000001	Weight decay = 0.00000001
Batch size = 10	Batch size = 10

The article "Deep-Learning-Based Cancer Profiles Classification Using Gene Expression Data Profile" was published in 2022. Journal: J Healthc Eng.

**Table 3:** Evaluation of proposed model based on training and testing.

Input parameters of classifier			Reduction in data			
313	(2, 35)	13	1.111	1.111	1.137	1.113
313	(2, 35)	33	1.138	1.119	1.333	1.131
313	(2, 35)	34	1.135	1.111	1.133	1.118
138	(1, 30)	33	0.019	0.010	0.131	0.009
138	(1, 30)	34	0.001	0.001	0.133	0.013
138	(1, 30)	13	0.017	0.004	0.138	0.014
138	(1, 30)	8	0.030	0.013	0.147	0.003
64	(1, 60)	64	0.017	0.001	0.138	0.003

**Table 4:** Performance comparison from various algorithms.

Precision		Recall	F1-score	Support
*Decision tree*				
0	0.38	0.50	0.43	6
1	0.88	0.81	0.85	27
Accuracy			0.76	0.33
Macro avg	0.63	0.66	0.64	33
Weighted avg	0.79	0.76	0.77	33
[[0.09 0.09]				
[0.15 0.67]]				

*Random forest*				
0	0.00	0.00	0.00	6.
1	0.82	1.00	0.90	27
Accuracy			0.82	33
Macro avg	0.41	0.50	0.45	33
Weighted avg	0.67	0.82	0.74	33
[[0. 0.18]				
[0. 0.82]]				

*Gaussian naive bayes*				
0	1.00	0.17	0.29	6
1	0.84	1.00	0.92	27
Accuracy			0.85	33
Macro avg	0.92	0.58	0.6	33
Weighted avg	0.87	0.85	0.80	33
[[0.03 0.15]				
[0. 0.82]]				

*Gradient descent (logistic)*				
0	0.62	0.83	0.71	3
1	0.96	0.89	0.92	27
Accuracy			0.88	33
Macro avg	0.79	0.86	0.82	33
Weighted avg	0.90	0.88	0.89	33
[[0.15 0.03]				
[0.09 0.73]]				

*Gradient descent (hinge)*				
0	0.00	0.00	0.00	6
1	0.82	1.00	0.90	27
Accuracy			0.82	33
Macro avg	0.41	0.50	0.45	33
Weighted avg	0.67	0.82	0.74	23
[[0. 0.18]				
[0. 0.82]]				

*Support vector machines*				
0	0.80	0.67	0.73	6
1	0.93	0.96	0.95	27
Accuracy			0.91	33
Macro avg	0.86	0.81	0.84	33
Weighted avg	0.91	0.91	0.91	33
[[0.12 0.06]				
[0.03 0.79]]				

*MLP (Adam)*				
0	0.18	1.00	0.31	6
1	0.00	0.00	0.00	27
Accuracy			0.18	33
Macro avg	0.09	0.50	0.15	33
Weighted avg	0.03	0.18	0.06	333
[[0.18 0. ]				
[0.82 0. ]]				

*MLP (LBFGS)*				
0	0.00	0.00	0.00	6
1	0.82	1.00	0.90	27
Accuracy			0.82	33
Macro avg	0.41	0.50	0.45	33
Weighted avg	0.67	0.82	0.74	33
[[0. 0.18]				
[0. 0.82]]				

**Table 5:** Accuracy calculation of the proposed system.

Precision		Recall	F1-score	Support
Class negative	0.85	0.92	0.88	12
Class negative	0.88	0.78	0.82	9
Avg/total	0.86	0.86	0.86	21
Accuracy is: 98.97%				

## Data Availability

The data that support the findings of this study are available upon request from the corresponding author.
